This article has been retracted.

# A Study of Feature Construction Based on Least Squares and RBF Neural Networks in Sports Training Behaviour Prediction

**DOI:** 10.1155/2022/5034081

**Published:** 2022-03-07

**Authors:** Chunyan Qiu, Changhong Su, Xiaoxiao Liu, Dian Yu

**Affiliations:** ^1^College of Sports and Physical Education, Shandong Sport University, Rizhao 276827, Shandong, China; ^2^Sports Section, Guangshui Road Primary School, Qingdao 266100, Shandong, China; ^3^Faculty of Engineering and Technology, School of Engineering, Liverpool John Moores University, Liverpool, UK

## Abstract

This paper examines the problem of athletes' training in sports, exploring the methods and means by which athletes can perform difficult movements in which they normally make minor training errors in order to achieve better competition results and placements. To this end, we test the explanatory and predictive effects of a theoretical model starting with planned behaviour and then use exercise planning, self-efficacy, and support as variables to develop a partial least squares regression model of sports to improve the explanation and prediction of sporting athletes' intentions and behaviour. An improved RBF network-based method for player behaviour prediction is proposed. On the basis of the RBF analysis, the number of layers and the number of neurons in the hidden layer of the network are adjusted and optimised, respectively, to improve its generalisation and learning abilities, and the athlete behaviour prediction model is given. The results demonstrate the advantages of the improved algorithm, which in turn provides a more scientific approach to the current basketball training.

## 1. Introduction

What if, after countless hours of practice, a sportsperson realises that there is only a 50% chance of successfully completing one of the most difficult manoeuvres of the entire competition and that the athlete might miss the most important and critical moment of the competition? What does the athlete do when faced with these potential threats? Many scholars have suggested adjusting one's breathing to regulate one's emotions, controlling oneself from thinking that the action has a high probability of being wrong, adjusting one's mental state so that he can perform the technique successfully, etc. [1]. However, numerous studies have shown that the use of intentions alone is not a good predictor of behaviour change. Action plans and coping plans are self-adjustment strategies. In many domains, behavioural intentions are supported after planning and execution as a motivation is received. The addition of a theory of planned behaviour appears to be the most appropriate as the theory of planned behaviour lacks sequential structure. It has also been found that when using behavioural interventions, research has not found an effect on behaviour by making implementation intentions, and on the basis of existing research, planning is more important as a mediating variable, and this paper will continue to examine and explore the forecasting effects of planning as an intermediate variable [2].

Currently, most of the research studies in the field of video-based motion human analysis are focused on motion behaviour recognition, but not on motion behaviour prediction. However, in real life, prediction of human movement based on the video is more valuable than behaviour recognition [3]. The public security department can be alerted to the predicted criminal behaviour in time to take corresponding measures. This not only reduces the amount of manpower and material and financial resources spent on security investigations but also provides effective prevention of sudden crime [4]. In the sports sector, a comprehensive set of video-based human movement prediction technologies can be used to accurately capture the game data of some of the best teams during sports training and to create a predictive discriminator for each athlete [5, 6].

The contributions of this paper are as follows:

  We start from the planned behaviour to test the interpretation and prediction effect of the theoretical model and then take the exercise plan, self-efficacy, and support as variables to establish the partial least squares regression model of sports, so as to improve the interpretation and prediction of aerobics athletes' intention and behaviour.
  We propose a team member behaviour prediction method based on the improved RBF network. The RBF network is analyzed. Based on the RBF analysis, the number of network layers is adjusted and optimized to improve its generalization and learning abilities, and the athlete behaviour prediction model is given.
  Based on the analysis of the sports competition video, the improved RBF is used to predict the athletes' behaviour, and the prediction results are compared with the traditional prediction results. The results show that our algorithm has advantages.

## 2. Related Work

At present, the research of individual sports is mainly reflected in the movement recognition and analysis of athletes [7–9] using target detection and tracking technology, the moving target is extracted from the diving video, and the moving target is video synthesized. A motion recognition method based on the human contour curvature scale space template is proposed and applied to the motion recognition of players in tennis competition [10]. The movements of ice hockey and football players are analyzed and studied. The movement direction of players is identified by using the histogram of oriented gradient (HOG) and hidden Markov model (HMM) [11–13]. The player's gestures in the low-resolution tennis game video are recognized [14]. By tracking the key points of some body parts of ballet dancers, the dance trajectory is obtained, and the automatic analysis of dance movements is realized [15]. It realizes the recognition of four swimming strokes in the swimming competition video.

In recent years, as research on individual sports analysis has matured so has research on multiplayer team sports [16]. Zhong and Xiao [17] investigated the patterns of passes that help to score goals in football and used multiscale analysis to cluster passes hierarchically and to mine the pattern categories of passes; Chen et al. [18] classified the trajectory and landing point of the ball as special cases in tennis and used an improved Bayesian network to fuse these two features. Li and Zhang [19] proposed a method for two-sided team possession situations, which is based on the ball position and the detection of the interplay, the local minima of the ball motion trajectory velocity of a player's possession start, the local minima of the ball position coordinates, the player's position, and the ball acceleration start point to infer the player's touch point. Li et al. [20] integrated a variety of information on the pitch in the ritual to achieve automatic analysis of football game tactics.

## 3. Development of a Regression Model for Sports Training

Simplify the data structure and correlation analysis of bivariate variables, greatly facilitating multivariate data analysis [21]. It uniquely suits to deal with small sample sizes and independent variables with significant multiple correlations between variables. However, the partial least squares regression model can be expressed as the original regression equation for all variables. The partial least squares regression method selects principal components that also include all variables and does not fully address the more severe multivariate correlations, especially in the case of some independent variables and small sample conditions [22].

In this paper, data from sports athletes regarding physical training were used to conduct partial least squares regression modelling in terms of the explanatory and predictive power of three variables—exercise program, self-efficacy, and social support—on exercise intention and behaviour and their role in the intention-to-behaviour process. The subjects of this paper were 10 players of a sports team. The first group of variables was exercise planning, self-efficacy, and social support. In this study, social support consisted of two types, family social support and friend social support, which were not effective predictors of exercise intention. The second group of variables was the training performance indicators of the sport players, which were rotation, bending, and high jump. The raw data are shown in Table 1, and the correlation coefficient matrix is shown in Table 2.

The simple correlation matrix of these six variables shows that an exercise program and self-efficacy are positively correlated; work program and self-efficacy are negatively correlated with social support, and rotation, bending, and high jump are positively correlated.

The partial least squares regression model is calculated by presenting two components *t*_1_ and *t*_2_, which have a cross-validity of *Q*_2_^2^ = −0.1969. The regression equation for the standardised variable $\bar{y_{k}}$ on component *t*_1_ in this paper is as follows:

(1) $$\begin{array}{c} \bar{y_{k}}=r_{1k}t_{1}+r_{2k}t_{2},k=1,2,3. \end{array}$$

The resulting partial least squares regression equation for component *t*_1_ is

(2) $$\begin{array}{c} \bar{y_{k}}=r_{1k}\left(w_{11}^{*}\bar{x_{1}}+w_{21}^{*}\bar{x_{2}}+w_{31}^{*}\bar{x_{3}}\right)+r_{2k}\left(w_{21}^{*}\bar{x_{1}}+w_{31}^{*}\bar{x_{2}}+w_{32}^{*}\bar{x_{3}}\right)\\ =\left(r_{1k}w_{11}^{*}+r_{2k}w_{12}^{*}\right)\bar{x_{1}}+\left(r_{1k}w_{21}^{*}+r_{2k}w_{22}^{*}\right)\bar{x_{2}}+\left(r_{1k}w_{31}^{*}+r_{2k}w_{32}^{*}\right)\bar{x_{3}}. \end{array}$$

The calculations for *r*_*h*_=(*r*_*h*1_, *r*_*h*2_, *r*_*h*3_) are

(3) $$\begin{array}{c} \bar{y_{1}}=-0.07\bar{x_{1}}-0.489\bar{x_{2}}-0.122\bar{x_{3}},\\ \bar{y_{2}}=-0.15\bar{x_{1}}-0.5244\bar{x_{2}}-0.054\bar{x_{3}}. \end{array}$$

The following equation is obtained by reducing the normalized variables $\bar{y_{k}},\bar{x_{k}}\left(k=1,2,3\right)$ to *y*_*k*_, *x*_*k*_(*k*=1,2,3), respectively:

(4) $$\begin{array}{c} y_{1}=47.97-0.07x_{1}-0.87x_{2}-0.99x_{3},\\ y_{2}=612.71-0.39x_{1}-10.2477x_{2}-0.71x_{3},\\ y_{3}=183.949-0.13x_{1}-2.49x_{2}-0.01x_{3}. \end{array}$$

## 4. RBF Radial Neural Network Prediction Model

From a structural point of view, the RBF nerve network consists of three layers: an input layer, an implicit layer, and an output layer. The number of nodes in this layer is determined by the actual number of input variables; the number of nodes in the implicit layer is difficult to determine and is determined by the complexity of the problem being described [23]; the output layer is used to output the results of the input and output processing of the system. In the RBF neural network, the transformation from the input space to the hidden space is a nonlinear transformation, and the transformation from the hidden layer to the input layer is a linear transformation. Assuming that the RBF neural network has only one hidden unit [24], the training sample of the RBF neural network can be expressed as {*X*_*n*_, *d*_*n*_}(*n*=1,2, ⋯, *N*). In this formula, *X*_*n*_=[*x*_*n*1_, *x*_*n*2_, ⋯,*x*_*nM*_]^T^(*n*=1,2, ⋯, *N*) is the sample input; *d*_*n*_(*n*=1,2, ⋯, *N*) is the desired sample output, and the corresponding actual output is *Y*_*n*_(*n*=1,2, ⋯, *N*); the radial basis function *φ*(*X*, *t*_*i*_) is the output of the *i*th hidden unit, and [*t*_*i*1_, *t*_*i*2_, ⋯,*t*_*im*_, ⋯,*t*_*iM*_]^(*i*=1,2, ⋯,*I*)^ is the centre of the basis function; *w*_*i*_(*i*=1,2, ⋯, *I*) is the connection weight between the *i*th hidden unit and the output unit.

The topology of a specific single-output RBF network is shown in Figure 1.

When the network input training sample is *X*_*n*_, the actual output of the network can be expressed by the following equation:

(5) $$\begin{array}{c} Y\left(X_{n}\right)=\sum_{i=1}^{\varepsilon }w_{i}\varphi \left(X,t_{i}\right). \end{array}$$

Currently, there are many RBF functions in the field of RBF neural networks, the most common of which are the Gaussian function, the multiple quadratic function, and the thin-slab spline function.

The purpose of data normalisation is to transform all data to values in the range [0, 1] to make subsequent calculations more convenient [25]. The data normalisation formula is

(6) $$\begin{array}{c} X=\frac{x-x_{\min}}{x_{\max}-x_{\min}}. \end{array}$$

The network parameters are updated by the following equation:

(7) $$\begin{array}{c} v_{i}=v_{i-1}+K_{i}e_{i},\\ K_{i}\left(zxn_{y}\right)=P_{i-1}B_{i}{\left[R_{i}+B_{i}^{T}P_{i-1}B_{i}\right]}^{-1},\\ P_{i}=\left[I_{zxz}-K_{i}B_{i}^{T}\right]P_{i-1}+q_{0}I_{zxz}. \end{array}$$

In the above equation, *v*_*i*_=[*w*_0_^*i*^, *w*_1_^*i*^, *c*_1_^*i*^, *δ*_1_^*i*^, ⋯,*w*_*K*_^*i*^, *c*_*K*_^*i*^, *σ*_*K*_^*i*^]^T^ represents the state of the parameter shown for the *i*th sample after it has entered the network.

The calculation is carried out for all hidden node outputs *σ*_*k*_=(*o*_*k*1_^*i*^, ⋯, *o*_*kj*_^*i*^, ⋯, *o*_*kn*_*y*__^*i*^),  *i*=1 ⋯ *N*, *k*=1, ⋯, *K*, *j*=1, ⋯, *n*_*y*_, and ‖*o*_*j*,max_^*i*^‖=max(‖*o*_1,*j*_^*i*^‖, ‖*o*_2,*j*_^*i*^‖, ⋯, ‖*o*_*K*,*j*_^*i*^‖, (*j*=1, ⋯, *n*_*y*_). The specific normalized output vector formula is

(8) $$\begin{array}{c} r_{kj}^{i}=\frac{\left\|o_{k,j}^{i}\right\|}{\left\|o_{j,\max}^{i}\right\|}\;\left(k=1,\cdots K\right). \end{array}$$

If all *r*_*kj*_^*i*^ < *ε*_2_ are established, then the *k*th hidden node can be deleted.

## 5. Experimentation and Analysis

In order to verify the effectiveness of the method, we experimented on an Intel Core 2 T6500 PC with 3 G RAM, implemented using VVC++6.0 with the OpenCV vision library programming [26]. To train the FSAMME-based head state classifier, we manually intercepted 800 head images from 100 basketball game videos, 100 images from each class. A typical training sample is shown in Figure 2. In addition, 100 nonhead images were intercepted as a negative example training set, consisting mainly of local stadium background blocks and blocks of other body parts of the players.  Figure 3 shows the relationship between the relative size (ratio to sample side length) of the small square area extracted from the training sample and the recognition accuracy. In the training process, we set *τ*_accuracy _ of the head image detection classifier to 0.9, the learning rate *τ*_rate _ to 0.1, and *τ*_accuracy _ of the nonhead image detection classifier to 0.4. We selected another 400 head images as the test set, 80 images of each class, and the experimental results are shown in Table 3.

As can be seen from Table 3, the misjudgements were mainly in the discrimination of two adjacent head poses. This is mainly due to the low resolution of the head image in the basketball game video, the interference of motion blur and noise, and the similarity of the adjacent head postures themselves. From the experimental results, it can be seen that the covariance descriptor, which incorporates a variety of underlying features, is well adapted to the above situation and achieves satisfactory experimental results, with the average recognition rate of various head poses.

In order to verify that the covariance descriptor can improve the accuracy of head state recognition after fusing the original underlying features, we have selected a subset of feature vectors in the section for comparison experiments, respectively, and the experimental results are colour features, gradient features, texture features, colour-gradient features, colour-texture features, gradient-texture features, and colour-gradient-texture features, as shown in Figure 4.

In addition, we also experimented with the method in this article in the case of partial occlusion of the player's head. Test cases were manually occluded from the top, bottom, left, and right directions, with each direction taking up 10%, 20%, 30%, 40%, and 50% of the total head image area, shown in Figure 5.

As can be seen from the graph, the accuracy of head pattern recognition is generally higher when the left and right occlusion occurs than when the top and bottom occlusion occurs. When the occlusion rate is reached, the lowest upper occlusion recognition rate is also higher than the best right occlusion recognition rate by a close margin. It can be seen that the method in this paper also achieves better results when dealing with partial occlusion.

Finally, the method is compared with two state-of-the-art methods for low-resolution cephalosporin recognition. As can be seen from Table 4, this method outperforms the other two methods in terms of average head pattern recognition rate.

## 6. Conclusions

The above analysis shows that the RBF neural network has strong generalization and learning abilities in dealing with the prediction of nonlinear problems, and the above construction shows that the algorithm proposed in this paper has more advantages and accuracy in the prediction of sports behaviour, thus proposing a new scientific training method for the scientific training of current sports.

## Figures and Tables

**Figure 1:** Topology of a single-output RBF network.

**Figure 2:** Typical training sample of the head state detection classifier.

**Figure 3:** Accuracy of head pattern recognition versus relative size of small areas.

**Figure 4:** Comparison of recognition rates for different types of original feature fusion.

**Figure 5:** Average head state recognition in different occlusion situations.

**Table 1:** Physical training data.

No.	Exercise program	Self-efficacy	Social support	Rotate	Bend	High jump
1	91	36	50	5	162	60
2	89	37	52	2	110	60
3	93	38	58	12	101	101
4	63	35	62	12	105	37
5	89	35	46	13	155	58
6	82	36	56	4	101	42
7	67	34	60	6	125	40
8	76	31	74	15	200	40
9	54	33	56	17	251	250
10	69	34	50	17	120	38

**Table 2:** Correlation coefficient matrix.

	*x*_1_	*x*_2_	*x*_3_	*y*_1_	*y*_2_	*y*_3_
*x*_1_	1	0.8702	−0.3658	−0.3897	−0.4931	−0.2263
*x*_2_	0.8702	1	−0.3529	−0.5522	−0.6456	−0.1915
*x*_3_	−0.3658	−0.3529	1	0.1506	0.225	0.0349
*y*_1_	−0.3897	−0.5522	0.1506	1	0.6957	0.4958
*y*_2_	−0.4931	−006456	0.225	0.6957	1	0.6692
*y*_3_	−0.2263	−0.1915	0.0349	0.4958	0.6692	1

**Table 3:** Results of the head state recognition experiment.

Degrees	0	45	90	135	180	225	270	315
0	0.98	0.01	0	0	0	0	0	0.01
45	0.01	0.96	0.02	0	0	0	0	0.01
90	0	0.02	0.95	0.01	0	0.01	0	0.01
135	0	0.01	0.02	0.95	0	0.01	0	0.01
180	0	0	0	0	0.99	0.01	0	0
225	0	0	0	0.01	0	0.97	0.02	0
270	0	0.01	0	0	0	0.01	0.96	0.02
315	0.02	0	0	0	0	0.01	0.01	0.96

**Table 4:** Comparison with two existing methods in terms of average recognition rate.

Method	Method in this paper	Orozco	Siriteerakul
Average identification	96.5%	71.7%	78.6%
accuracy			

## Data Availability

The datasets used during the current study are available from the corresponding author upon reasonable request.
